The article "MicroRNA‐520c enhances cell proliferation, migration, and invasion by suppressing IRF2 in gastric cancer" was retracted in 2022. Reasons: duplicated images; signs of a paper mill; concerns about the data.

# MicroRNA‐520c enhances cell proliferation, migration, and invasion by suppressing IRF2 in gastric cancer

**DOI:** 10.1002/2211-5463.12142

**Published:** 2016-10-31

**Authors:** Ying‐ru Li, Li‐qiang Wen, Yang Wang, Tai‐cheng Zhou, Ning Ma, Ze‐hui Hou, Zhi‐peng Jiang

**Affiliations:** ^1^ Department of GastroenterologyHernia and Abdominal Wall SurgeryThe Sixth Affiliated Hospital of Sun Yat‐Sen UniversityGuangzhouChina; ^2^ Department of Gastrointestinal SurgerySun Yat‐Sen Memorial HospitalSun Yat‐Sen UniversityGuangzhouChina; ^3^ Department of General SurgeryShenzhen Hospital of Armed Police Frontier CorpsChina

**Keywords:** cell mobility, cell proliferation, gastric cancer, interferon regulatory factor 2, microRNA‐520c

## Abstract

Dysregulation of microRNA (miRNA) is actively involved in the development and progression of gastric cancer (GC). MiR‐520c was previously found to be overexpressed in GC specimens and cells. However, the clinical significance of miR‐520c and its biological function in GC remain largely unknown. Here, we found that miR‐520c expression in GC tissues was significantly increased compared to normal adjacent gastric tissues. Its increased level was prominently correlated with poor clinical parameters and prognosis of GC patients. Accordingly, the expression of miR‐520c was obviously elevated in GC cell lines as compared with gastric epithelial cells. Overexpression of miR‐520c in N‐87 cells significantly increased the proliferative ability, migration, and invasion of cancer cells, while miR‐520c silencing suppressed MKN‐45 cell proliferation, migration, and invasion *in vitro*. Mechanically, miR‐520c inversely regulated interferon regulatory factor 2 (IRF2) abundance in GC cells. Herein, IRF2 was found to be a downstream target of miR‐520c in GC. Furthermore, IRF2 was down‐regulated in GC tissues compared to nontumor tissues. An inverse correlation between IRF2 and miR‐520c expression was observed in GC cases. Taken together, miR‐520c may serve as a prognostic predictor and a therapeutic target for GC patients.

**Abbreviations**
GC: gastric cancer
HCC: hepatocellular carcinoma
IRF2: interferon regulatory factor 2
TNM: tumor‐node‐metastasis

MicroRNA (miRNA), a group of small noncoding RNA interacting with the 3′‐UTR of targeted mRNA, inhibited the expression of target genes by contributing to the degradation or translational inhibition of target mRNA 1. They have been found to be actively involved in various biological processes 2, 3 including cell proliferation, apoptosis, differentiation, and movement. Emerging studies showed that abnormal expression and function of miRNA have found to play important roles in the initiation and progression of human malignancies 4, 5, 6. miRNA have also been demonstrated to be promising biomarkers and therapeutic targets of gastric cancer (GC) 7, 8, 9. Investigating the expression and biological function of miRNA in GC will contribute to the identification of novel biomarkers and therapeutic targets for GC patients.

Recently, microRNA‐520c was found to play important roles in various human cancers including diffuse large B‐cell lymphoma 10, breast cancer 11, fibrosarcoma 12, and hepatocellular carcinoma (HCC) 13. Study of breast cancer showed that miR‐520c could promote cancer cell migration and invasion *in vitro* and *in vivo* by suppression of CD44 14. And expression of miR‐520c increased proliferation, migration, and invasion of HCC cells *in vitro* 13. However, miR‐520c abrogated both *in vitro* cell invasion and *in vivo* intravasation of highly invasive MDA‐MB‐231 cells 11, indicating that miR‐520c functions as a tumor suppressor in estrogen receptor‐negative breast cancer. Previously, Yao *et al*. 15 analyzed the expression profile of microRNA in GC specimens from Chinese patients and miR‐520c‐3p was significantly up‐regulated in GC. Moreover, the expression of miR‐520c was markedly increased in MKN‐45 cells compared to cancer stem cells 16. However, the clinical significance and biological role of miR‐520c in GC remain poorly known.

Here, we confirmed that the expression of miR‐520c was overexpressed in GC tissues and cells. High expression of miR‐520c was correlated with poor clinicopathological features and reduced survival of GC patients. Our data showed that miR‐520c promoted the proliferative and metastatic ability of GC cells *in vitro*. Moreover, Interferon regulatory factor 2 (IRF2) was identified as a downstream target of miR‐520c in GC.

## Materials and methods

### Clinical tissues

Clinical specimens were collected from 90 patients with histologically diagnosed GC in The Sixth Affiliated Hospital of Sun Yat‐Sen University. No patients had received any chemotherapy or radiotherapy before surgical treatment. All clinical specimens were collected and used after obtaining informed consent from each patient enrolled in this study. All specimens were stored in liquid nitrogen for further investigation. The protocol involving clinical specimens in this study was approved by the Research Ethics Committee of Sun Yat‐Sen University.

### Cell culture and transfection

Human GC cell lines including N‐87, SGC‐7901, AGC, SNU‐16, and MKN‐45, and human gastric epithelial cells (GES‐1) were obtained from American Type Culture Collection (Manassas, VA, USA). These cells were cultured in Dulbecco's modified Eagle's medium (DMEM) with 10% FBS, 100 U·mL^−1^ penicillin, and 100 mg·mL^−1^ streptomycin. All cell cultures were maintained in humidified cell incubator with 5% CO_2_ at 37 °C.

miR‐520c mimic (HmiR0327‐MR04), miR‐520c inhibitor (HmiR‐AN0598‐AM04), and the corresponding control vectors (CmiR0001‐MR04; CmiR‐AN0001‐AM04) were bought from Genecopoeia (Guangzhou, China) and were then transfected into GC cells with lippofectamine 2000 following the manufacturer's protocol.

### Quantitative real‐time RT‐PCR

Total RNA from GC cells was extracted by miRNeasy Mini Kit (Qiagen, Hilden, Germany) and total RNA from GC tissues were extracted with Trizon reagent (Ambion; Thermo Scientific, Shanghai, China). miR‐520c levels in these samples were assayed using TaqMan MicroRNA assays based on the manufacturer's protocol (Applied Biosystems, Carlsbad, CA, USA). The primers for miR‐520c and U6 were obtained from Genecopoeia. U6 was employed as the internal control for miR‐520c.

### Luciferase reporter assay

To investigate whether miR‐520c could interact with the 3′‐UTRs of IRF2, wild‐type (wt) 3′‐UTR of IRF2 predicted to interact with miR‐520c or the mutant (mt) IRF2 3′‐UTR was amplified. Then, the wt 3′‐UTR of IRF2 or mt 3′‐UTR of IRF2, and miR‐520c mimic were cotransfected into GC cells by lippofectamine 2000. Forty‐eight hours after cotransfection, the cells were lysed and assayed using Dual‐Luciferase® Reporter Assay Kit (Promega, Madison, WI, USA) based on the manufacturer's instructions.

### Wound healing assay

Gastric cancer cells transfected with corresponding vectors were seeded in six‐well plates to form the single confluent cell layer. The wounds were made with 100 µL tips in the confluent cell layer. About 0 and 12 h after wound scratching, the width of wound was photographed with phase‐contrast microscope.

### Migration and invasion assay

The migratory and invasive ability of GC cells were evaluated with Transwell chambers (BD Biosciences, Franklin Lakes, NJ, USA). GC cells (5–10 × 10^4^) suspended in 100 µL serum‐free medium were seeded into the upper chamber, and the lower chamber was filled with 20% FBS to induce GC cells migrating or invading through the membrane. Matrigel (1 : 6 dilution; Becton Dickinson Labware, Bedford, MA, USA) was added on the upper chamber for invasion assay. Twenty‐four hours later, cells that migrated or invaded across the Transwell membrane were stained with crystal violet and the cell number was counted under microscope.

### Proliferation assays

For cell proliferation, GC cells that were treated with miR‐520c mimic or inhibitor were seeded into 96‐well plates (1.5 × 10^3^ cells per well). Twenty‐four, 48, 72, and 96 h after transfection, the cell proliferation assay was performed by the addition of 10 μL of cell counting kit 8 (CCK8) solution (Beyotime, Shanghai, China) to each well, followed by incubation at 37 °C for 2 h. Absorbance was measured at a wavelength of 490 nm using a microplate reader (Flexstation III ROM V2.1.28, Molecular Devices, Sunnyvale, CA, USA).

### Western blot

Before protein extraction, GC cells were washed with PBS to remove the culture media. Cellular proteins were obtained from GC cells using RIPA lysis buffer and the protein concentrations were measured with BSA method. Thirty micrograms of cellular proteins were separated by 10% SDS/PAGE, and were transferred to polyvinylidene fluoride (PVDF) membrane (Millipore, Bedford, MA, USA). After blocking with 5% nonfat milk at room temperature for 1 h, the membranes were probed with primary antibodies at 4 °C overnight. Then, the membranes were incubated with corresponding secondary antibodies at room temperature for 2 h. The primary antibodies used in this study included: IRF2 (Abcam, Cambridge, UK) and GAPDH (Abcam).

### Immunohistochemistry

Before immunohistochemistry (IHC) staining, GC and nontumor tissues were fixed with 4% formalin and embedded with paraffin. Then, the embedded tissues were cut into 4‐μm‐thick sections and IHC staining following standard protocol to evaluate the expression level of IRF2 (Abcam) in GC and nontumor tissues was carried out. The percentage of positive tumor or gastric cells was graded as per the following criteria: 0, less than 10%; 1, 10–30%; 2, 31–50%; 3, more than 50%.

### Statistical analysis

All quantitative data were presented as the mean ± SEM. Statistical analyses including Pearson chi‐squared test, a two‐tailed Student's *t* test, ANOVA, Kaplan–Meier method and the log‐rank test, Cox regression analysis, and Spearman's correlation analysis were performed with graphpad prism 6 (GraphPad Software Inc., San Diego, CA, USA). *P* < 0.05 was considered to be statistically significant.

## Results

### miR‐520c expression is increased in GC tissues and cells

To examine the expression status of miR‐520c in GC, quantitative real‐time RT‐PCR was performed for 90 pairs of GC tissues and adjacent nontumor tissues. Our results showed that GC tissues had significant increased expression levels of miR‐520c compared with adjacent nontumor tissues (*P* < 0.05, Fig. 1A). Then, we compared the expression level of miR‐520c between GC cells and gastric epithelial cells. Compared with GES‐1 cells, the expression levels of miR‐520c in all five GC cell lines including N‐87, SGC‐7901, AGS, SNU‐16, and MKN‐45 was significantly elevated (*P* < 0.05, Fig. 1B). These indicate miR‐520c probably plays an oncogenic role in GC.

**Figure 1:** The expression of miR‐520c in GC. (A) Significant increased expression of miR‐520c was observed in GC tissues. *n* = 90, *P < 0.05 by *t* test. (B) The expression levels of miR‐520c in GC cells (N‐87, SGC‐7901, AGS, SNU‐16, and MKN‐45), as well as in GES‐1 cells. *n* = 3 repeats with similar results, *P < 0.05 versus GES‐1 by ANOVA. Values are mean ± SEM.

### High expression of miR‐520c correlates with poor clinical features and prognosis of GC patients

To clarify the clinical significance and prognostic value of miR‐520c in GC, all patients were divided into two groups: miR‐520c low group and miR‐520c high group. As shown in Table 1, compared with those with low expression of miR‐520c, patients with high expression of miR‐520c had more lymph node metastasis (*P* = 0.019) and advanced tumor‐node‐metastasis (TNM) stage (*P* = 0.018). Furthermore, Kaplan–Meier analysis showed that patients with high expression of miR‐520c showed significantly reduced overall survival and disease‐free survival (*P* = 0.012 and *P* = 0.015, respectively, Fig. 2). In addition, the Cox‐regression analysis showed that miR‐520c expression was an independent factor for predicting the survival of GC patients (*P* < 0.05, Table 2). These indicate that miR‐520c is actively involved in the development and progression of GC.

**Table 1:** The correlation between miR‐520c and clinicopathologic features in gastric cancer. TNM, tumor‐node‐metastasis

Characteristics	Total	miR‐520c expression		*P*
		High (45)	Low (45)	
Age (years)				
<65	39	20	19	0.832
≥65	51	25	26	
Sex				
Male	70	34	36	0.612
Female	20	11	9	
Tumor differentiation				
I, II	42	17	25	0.091
III, IV	48	28	20	
Size (cm)				
<5	42	18	24	0.143
≥5	48	27	21	
Invasive depth				
Mucosa to muscularis propria	11	4	7	0.334
Adventitia to adjacent structure	79	41	38	
Lymph nodes metastasis				
≤2 regions	39	14	25	0.019^a^
>2 regions	51	31	20	
Distant metastasis				
No	68	31	37	0.141
Yes	22	14	8	
Venous infiltration				
Absent	67	30	37	0.091
Present	23	15	8	
TNM stage				
I, II	37	13	24	0.018^a^
III, IV	53	32	21	

a Statistically significant.

**Figure 2:** The prognostic predicting value of miR‐520c in GC. Compared with those of low miR‐520c level (*n* = 45), patients with high miR‐520c expression (*n* = 45) had significantly decreased overall survival and disease‐free survival. *P* < 0.05 by Kaplan–Meier method and the log‐rank test.

**Table 2:** Multivariate analyses of factors associated with survival. TNM, tumor‐node‐metastasis

Variables	Overall survival			Disease‐free survival		
	HR	95% CI	*P*	HR	95% CI	*P*
Tumor differentiation	0.82	(0.33–2.00)	0.658	0.77	(0.31–1.90)	0.567
Lymph nodes metastasis	2.35	(1.25–4.41)	0.008^a^	2.43	(1.30–4.59)	0.006^a^
Distant metastasis	7.89	(4.58–13.61)	<0.001^a^	9.41	(5.49–16.16)	<0.001^a^
TNM stage	1.61	(1.01–2.59)	0.049^a^	1.77	(1.10–2.86)	0.019^a^
miR‐520c expression	0.44	(0.22–0.86)	0.016^a^	0.43	(0.27–1.02)	0.038^a^

a Statistically significant.

### miR‐520c facilitates the proliferation, migration and invasion of GC cells

Next, we explored whether miR‐520c could modulate the proliferation, migration and invasion of GC cells. N‐87 cells that showed the lowest level of miR‐520c in five GC cell lines were employed for gain‐of‐function experiments. Transfection of miR‐520c mimic into N‐87 cells significantly increased the expression level of miR‐520c (*P* < 0.05, Fig. 3A). Proliferation assays indicated that the proliferative ability of N‐87 cells was evidently enhanced 72 h after transfection (*P* < 0.05, Fig. 3B). The wound healing assays showed that the migration of N‐87 cells was significantly increased after miR‐520c overexpression (*P* < 0.05, Fig. 3C), and Transwell assays demonstrated that overexpression of miR‐520c prominently promoted the migration and invasion of N‐87 cells (*P* < 0.05, respectively, Fig. 3D). MKN‐45 cells that showed the highest level of miR‐520c in five GC cell lines were employed for loss‐of‐function experiments. On the contrary, miR‐520c inhibitor significantly decreased the expression level of miR‐520c in MKN‐45 cells (*P* < 0.05, Fig. 4A). Subsequently, miR‐520c silencing significantly inhibited the proliferation, migration, and invasion of MKN‐45 cells (*P* < 0.05, respectively, Fig. 4B–D).

**Figure 3:** miR‐520c mimic promotes the proliferation, migration, and invasion of N‐87 cells. (A) miR‐520c mimic significantly increased the level of miR‐520c expression in N‐87 cells. *n* = 3 repeats with similar results, *P < 0.05 by *t* test. (B) CCK8 assays indicated that miR‐520c overexpression enhanced N‐87 cell proliferation. *n* = 3 repeats with similar results, *P < 0.05 by ANOVA. (C) miR‐520c overexpression potentiated the migration of N‐87 cells. *n* = 3 repeats with similar results. (D) miR‐520c overexpression promoted the migration and invasion of N‐87 cells. *n* = 3 repeats with similar results, *P < 0.05 by *t* test. Values are mean ± SEM.

**Figure 4:** miR‐520c inhibitor inhibits the proliferation, migration, and invasion of MKN‐45 cells. (A) miR‐520c inhibitor significantly decreased the expression of miR‐520c in MKN‐45 cells. *n* = 3 repeats with similar results, *P < 0.05 by *t* test. (B) iR‐520c silencing reduced the proliferative ability of MKN‐45 cells. *n* = 3 repeats with similar results, *P < 0.05 by ANOVA. (C) miR‐520c knockdown significantly decreased the migration of MKN‐45 cells. *n* = 3 repeats with similar results. (D) miR‐520c knockdown significantly suppressed the migration and invasion of MKN‐45 cells. *n* = 3 repeats with similar results, *P < 0.05 by *t* test. Values are mean ± SEM.

### IRF2 is a downstream target of miR‐520c

To disclose the underlying molecular mechanisms for the biological function of miR‐520c in GC cells, TargetScanHuman 7.1 (http://www.targetscan.org) was used to search for the downstream target of miR‐520c. IRF2, an oncosuppressor in GC 17, was recognized as a potential downstream target of miR‐520c. As shown in Fig. 5A, 3′‐UTR of IRF2 contained the putative bind sites for miR‐520c. Then, we performed luciferase assay to investigate whether miR‐520c could bind to the putative‐binding sites in the 3′‐UTR of IRF2. Overexpression of miR‐520c decreased the luciferase activity of wt IRF2 3′‐UTR (*P* < 0.05, Fig. 5B), while miR‐520c overexpression did not have any influence on the luciferase activity of mt IRF2 3′‐UTR (Fig. 5B). Accordingly, alteration of miR‐520c expression inversely regulated IRF2 abundance in GC cells (Fig. 5C). Therefore, these data indicate IRF2 is a direct downstream target of miR‐520c in GC.

**Figure 5:** miR‐520c binds to the complementary sequence in 3′‐UTR of IRF2. (A) The binding sites for miR‐520c in 3′‐UTR of IRF2. (B) Overexpression of miR‐520c decreased the luciferase activity of wt 3′‐UTR of IRF2, while alteration of miR‐520c had no effect on the luciferase activity of mutant 3′‐UTR of IRF2 in both N‐87 and SGC‐7901 cells. *n* = 3 repeats with similar results, *P < 0.05 by *t* test. (C) miR‐520c overexpression reduced while miR‐520c silencing increased the level of IRF2 protein in N‐87 and MKN‐45 cells, respectively. *n* = 3 repeats with similar results, *P < 0.05 by *t* test. Values are mean ± SEM.

### An inverse correlation between IRF2 and miR‐520c is observed in GC specimens

Gastric cancer and nontumor tissues were subjected to immunohistochemistry for IRF2 expression. IHC scores evaluation indicated that the expression of IRF2 in GC tissues was significantly lower than that in nontumor tissues (*P* < 0.05, Fig. 6A, B). Furthermore, miR‐520c high expressing tumors showed weak staining of IRF2, while miR‐520c low expressing tumors showed strong staining of IRF2 (Fig. 6A). Spearman's correlation analysis indicated that miR‐520c was strongly correlated with IRF2 expression in GC specimens (*r* = −0.634, *P* < 0.001, Fig. 6C).

**Figure 6:** The correlation between IRF2 and miR‐520c in GC tissues. (A) Representative immunohistochemical staining of IRF2 in GC and nontumor tissues. miR‐520c high expressing tumors showed weak staining of IRF2, while miR‐520c low expressing tumors showed strong staining of IRF2. Scale bar: 100 μm. (B) The expression of IRF2 was down‐regulated compared to nontumor tissues. *n* = 90, *P < 0.05 by *t* test. (C) An inverse correlation between IRF2 and miR‐520c expression was observed in GC tissues. *n* = 90, *P* < 0.05 by Spearman's correlation analysis. Values are mean ± SEM.

## Discussion

Emerging evidences have confirmed that miRNA are actively involved in the pathogenic process of GC 18. In addition, miRNA have been found to be critical regulators of the metastasis and epithelial–mesenchymal transition of GC cells 8. Due to the important roles of miRNA in GC, miRNA have been proposed as promising biomarkers and therapeutic targets of GC 18. In this study, miR‐520c was found to be significantly up‐regulated in GC tissues and cells as previously reported 15, 16. The high expression of miR‐520c in GC tissues conferred poor clinical features of GC patients including lymph node metastasis and advanced TNM stage. More importantly, elevated expression of miR‐520c was correlated with reduced overall survival and disease‐free survival of GC patients, and was found to be an independent factor for predicting the prognosis of GC patients. Therefore, miR‐520c plays an oncogenic role in GC and potentially serves as promising biomarker for the prognosis of GC patients.

Systemic metastasis is the important reason for the unsatisfactory prognosis of GC patients 19. Increased migratory and invasive ability of GC cells underlies the systemic metastasis of GC 19. Therefore, it is of great importance to elucidate the molecular mechanisms for the metastasis of GC cells. In this study, we found that miR‐520c promoted the migration and invasion of GC cells *in vitro*, suggesting that miR‐520c exerted a prometastatic role in GC. Moreover, invasive growth is a hallmark of human cancer and is a critical mechanism for cancer metastasis 20. Our results showed that miR‐520c enhanced the proliferative ability of GC cells. Taken together, these data demonstrate that miR‐520c functions as an oncomiR by promoting proliferation, migration, and invasion in GC cells.

Interferon regulatory factor 2 was initially found to inhibit the interferon‐inducible genes transcription in 1898 21. IRF2 functions as a tumor suppressor in HBV‐related HCC 22, while the oncogenic role of IRF2 was reported in some cancer cells 23, 24, 25. Therefore, the functions of IRF2 depends on cell type or context. Recently, IRF2 was reported to be down‐regulated and regulated by miR‐18a in GC. In this study, we found that miR‐520c negatively regulated the abundance of IRF2 in GC cells. And the expression of IRF2 in GC tissues was inversely correlated with miR‐520c expression. Moreover, we found that miR‐520c could directly interact with the 3′‐UTR of IRF2 using a luciferase reporter assay. These data indicate that IRF2 is a direct downstream target of miR‐520c in GC.

In all, this study demonstrates that miR‐520c expression is significantly overexpressed in GC tissues and cells. Increased expression of miR‐520c is correlated with adverse clinical features and poor prognosis of GC patients. In addition, miR‐520c promotes proliferation, migration, and invasion of GC cells. Furthermore, IRF2 is a direct downstream target of miR‐520c in GC. These data may result in the discovery of therapeutic candidates of GC.

## Conclusions

In summary, this study shows that the expression of miR‐520c is up‐regulated in GC tissues compared to matched noncancerous tissues. Furthermore, elevated expression of miR‐520c was observed in GC cells compared to gastric epithelial cells. Clinical data indicate that high expression of miR‐520c is evidently associated with poor prognostic features of GC. Notably, miR‐520c expression is an independent prognostic marker for predicting 5‐year overall and disease‐free survival of GC patients. Gain‐of‐function studies demonstrate that miR‐520c overexpression promotes proliferation, migration, and invasion of N‐87 cells. On the contrary, miR‐520c silencing inhibits MKN‐45 cell proliferation, migration, and invasion. Our data indicate that miR‐520c inversely regulates the abundance of IRF2 in GC cells. Herein, IRF2 is identified as a direct downstream target of miR‐520c. Furthermore, IRF2 expression is down‐regulated in GC tissues and it is inversely correlated with the levels of miR‐520c. This study reveals that miR‐520c may play a critical role in the tumor growth and metastasis of GC and may be a potential prognostic biomarker and therapeutic target for GC.

## Author contributions

YL, LW, YW, TZ, NM, and ZH carried out the cell biology and molecular biology experiments, participated in the sequence alignment, and drafted the manuscript. YL, LW and ZJ participated in the design of the study and performed the statistical analysis. ZJ conceived of the study, and participated in its design and coordination, and helped to draft the manuscript. All authors read and approved the final manuscript.
